RETRACTED

# A Mode of Intelligent Equipment Monitoring Optimization Based on Dynamic Programming Algorithm

**DOI:** 10.1155/2022/1569428

**Published:** 2022-03-18

**Authors:** Zhilei Zheng, Chuan Jiang

**Affiliations:** Department of Physical Education, Shandong University, Weihai 264200, China

## Abstract

With the continuous development of the national economy and scientific productivity, urban construction and people's living standards are also getting higher and higher. Although people enjoy increasingly convenient life, the demand for intelligence is getting higher and higher. Digital intelligent equipment has the functions of data collection, calculation and analysis, diagnostic and early warning, and communication functions. Analyze the status quo and existing problems of the development of intelligent equipment, as well as analyze and research key monitoring technologies in the use and development of digital intelligent equipment and provide optimal solutions for intelligent equipment hardware development requirements, software development, and model algorithms. Intelligent equipment monitoring is related to all aspects of people's livelihood, and its intelligent development is related to the public role in this field in the future. Accurate results of monitoring can provide data support for schools, research institutions, the public, and the government. At the same time, it is also an important basis for formulating social policies. At present, the commonly used monitoring method usually adopts time series algorithm. Through literature review, it is found that the algorithm has the problem of distortion of correct data, which affects the accuracy of monitoring results. Based on the above reasons, this article combines the wavelet function with the planning algorithm and proposes a dynamic programming algorithm, which removes the redundant monitoring data in turn and clusters the distortion monitoring data with the wavelet function, which improves the accuracy and computational efficiency of the algorithm and gives full play to the monitoring of intelligence. The simulation results using MATLAB show that the planning algorithm can eliminate 90% of redundant monitoring data and improve the extraction rate of characteristic monitoring data. At the same time, the accuracy of the planning algorithm reaches 95%, and the calculation time is less than 25 s, which is better than the static planning algorithm. Therefore, the dynamic programming algorithm can better utilize the intelligence, convenience, and efficiency of the equipment to optimize the monitoring model.

## 1. Introduction

Intelligent devices have been widely used in engineering technology, industrial production, social services, medicine, and human health, and they have had an important impact. Intelligent equipment monitoring is an important part of social public health. It is not only the guarantee of Chinese public health but also the basis for the improvement of national quality[1]. The integration of intelligent equipment and modern technology not only enhances the intelligence of monitoring but also realizes its own function optimization. Continuous and dynamic intelligent equipment monitoring and analysis of the public can help the government make health decisions and improve the disease resistance and physical quality of the public Beuchat et al. [2]. In the past, the public monitoring method was mainly planning algorithm. Although this algorithm can monitor the general health, it cannot carry out dynamic analysis, and the analysis results have some limitations. In addition, there are a lot of redundant data in intelligent equipment monitoring, which affects the monitoring results of college students [3]. At present, there are many researches on intelligent equipment device monitoring of college students, but the redundancy of monitoring data is also high, as shown in Figure 1. Therefore, the application of dynamic programming method in the optimal control of intelligent equipment has very important theoretical significance. At the same time, the large-scale application of intelligent devices needs more effective algorithms as support, so this study can provide more practical cases, which has very important practical significance.

RETRACTED

Some scholars such as Fortune et al. [4] also believe that the increasing intelligent characteristic data in the static programming algorithm will improve the intelligence of monitoring but reduce the accuracy of monitoring. Therefore, a dynamic programming algorithm is constructed and revised to improve the accuracy of the results [5]. As a processing method of comprehensive function, wavelet function can subcontract the content data into fragmented data groups, improve the processing capacity of initial data, and is widely used in the optimization of a large number of intelligent devices. However, it is not used in dynamic programming algorithm at present. Therefore, this article attempts to apply it to the dynamic programming algorithm and construct a new intelligent device optimization model, which aims to improve the data processing efficiency of intelligent devices and promote the development of intelligent devices. Dynamic programming algorithm is developed on the basis of static programming algorithm. It is to add time variables to the original algorithm and continuously combine the static programming algorithm. However, the fundamental difference between dynamic algorithm and static algorithm is to increase the coupling between different indexes and make the calculation results more continuous. At the same time, the improvement of coupling also increases the complexity of calculation and the incidence of redundant data. Based on the research of scholars at home and abroad, the integration of wavelet function and dynamic programming algorithm can use the subcontracting method of wavelet function to increase the data processing capacity of dynamic programming algorithm, reduce the occurrence rate of local extremum, and improve the accuracy of calculation results. Dynamic programming algorithm can continuously track intelligent devices without being affected by the increase of data volume. Therefore, the integration of wavelet function and dynamic programming algorithm has the advantage of comprehensive analysis and improves the processing capacity of calculation data. Based on the above reasons, this article combines the discrete wavelet function with the planning algorithm to construct a dynamic planning algorithm to optimize the health monitoring results of College Students' wearing devices [6]. Taking college students' physical health monitoring as an analysis case, this article improves the accuracy of the results, so as to better carry out intelligent health monitoring.

RETRACTED

## 2. Algorithm Description of Intelligent Health Monitoring Devices

The key of intelligent equipment monitoring is to quantify the relevant indicators in intelligent equipment devices, so as to lay a mathematical foundation for dynamic monitoring. Among them, height, weight, 50-meter run, 800-meter run (girls), and 1000-meter run (boys) have more wearing equipment [7], whereas there are relatively few data on vital capacity, standing long jump, sitting body flexion, sit ups, step test and pull-up, but the algorithm description of health monitoring data are required.

### 2.1. Intelligent Health Monitoring Process of College Students

Intelligent health monitoring of intelligent equipment devices includes three aspects: the data structure *x*_*i*_ in sports intelligent equipment devices, the impact of intelligence on health monitoring *x*_*j*_, and the dynamics *x*_*k*_ of health monitoring [8]. The data structure in the intelligent equipment device also includes the intelligent equipment device *x*_*i1*_, the proportion of different sports *x*_*i2*_, and the degree of cooperation between different sports *x*_*i3*_; similarly, the impact of intelligence on health monitoring include the promotion degree of intelligent technology to health monitoring *x*_*j1*_, the integration degree of intelligent technology and health monitoring *x*_*j2*_, and the promotion level of intelligent technology to health monitoring *x*_*j3*_; The dynamics of health monitoring include cooperation degree between cardiopulmonary monitoring, blood oxygen monitoring, blood pressure monitoring, and exercise monitoring *x*_*k1*_, cooperation between devices in different forms of intelligent technology *x*_*k2*_, and communication cooperation between different intelligent technologies *x*_*k3*_. According to the above analysis, college students' intelligent equipment monitoring involves many aspects, mainly including: height, weight, vital capacity, standing long jump, sitting forward flexion, 50 m running, sit ups, step test, pull up, 800 m running (girls), and 1000 m running (boys). At the same time, the collected monitoring data are massive (cloud monitoring data, a large number of applications of intelligent devices) and complex (there are a large number of unstructured monitoring data), which greatly reduces the accuracy of intelligent equipment monitoring in sports and cannot accurately reflect the intelligence of intelligent equipment devices. Because the mass and complexity are the inevitable trend of the development of intelligent equipment monitoring, a large amount of sports data of college students should be collected [9].

RETRACTED

### 2.2. Data Flow Description of College Students' Intelligent Equipment Monitoring

The stable wavelet function extracts the redundant data in college students' sports, makes discrete analysis on the intelligent equipment devices, and obtains the comprehensive monitoring data, so as to arrange the data in order to improve the accuracy of monitoring [10].

At the same time, the stable wavelet function uses discrete extraction to ensure the integrity of monitoring data in college students' sports and complete the single-phase characteristics of monitoring data in order. The specific monitoring data flow is described in Figure 2:

(1) Assuming that the intelligent equipment monitoring result is *A* and any intelligent equipment device *A*_*l*_ = {*a*_*1*_, *a*_*2*_,…, *a*_*n*_}, the relationship between *A* and each input monitoring data as follows:
  (1) $$\begin{array}{c} \sum_{l}^{n}A_{l}\overset{TS\left(\cdot \right)}{\underset{f\left(\cdot \right)}{\leftarrow }}{∲}_{n}\begin{array}{c} \overset{k-\text{means}}{\leftarrow }\\ \prod_{\text{indevie}}\sum_{i}^{n}x_{i}\overset{g\left(•\right)}{\underset{-g\left(•\right)}{⇄}}\sum_{j}^{n}x_{j}\overset{g\left(•\right)}{\underset{-g\left(•\right)}{⇄}}\sum_{k}^{n}x_{k} \end{array}, \end{array}$$
where *i,j,k* are natural numbers, *TS* (·) is the dynamic programming function, *f* (·) is the stable wavelet function, *G* (·) is the forward function between different input indexes, and - *G* (·) is the reverse function to complete the dynamic monitoring.
(2) Suppose that the monitoring result *a*_*l*_ of any sports event in intelligent health monitoring and the input *z* in the planning algorithm (data structure *x*_*i*_ in intelligent equipment devices [11], impact of intelligent technology on health monitoring *x*_*j*_, and dynamic *x*_*k*_ of health monitoring), *p* is the proportion of monitoring data (structured monitoring data >70%, semistructured monitoring data >70%, unstructured monitoring data >70%), *q* is the processing method of monitoring data distortion (reconstruction = 1, coefficient order = 2, quantification = 3, eigenvalue = 4, clustering = 4), then *c*_*l*_ is described as Inc_*l*_^*o*,*p*,*q*^, *o* ∈ (1,2,….., *n*), *p* ∈ (1,2,3,4), *q* ∈ (1,2,3,4). Among them, the logarithm in *In*(·) of *c*_*l*_ is used to avoid |*∞*| or extreme value 0, so as to ensure the effectiveness of the calculation results. The monitoring results of any sports are shown in Figure 2.
(3) The data structure *x*_*i*_ in devices, the impact of intelligence on health monitoring *x*_*j*_, and the dynamic *x*_*k*_ of health monitoring adopt the fusion function *f*(*x*) and propose the redundant monitoring data in college students' sports. The calculation formula of the function is as follows:
  (2) $$\begin{array}{c} \varphi \left(x\right)=\frac{\left[\bar{\bar{\left(\sum_{i=1}^{n}\alpha_{1}x_{i}+\sum_{j=1}^{n}\alpha_{2}x_{j}+\sum_{k=1}^{n}\alpha_{2}x_{k}\right)}}+\xi \right]}{\sum_{i,j,k=1}^{n}\left(x_{i}+x_{j}+x_{k}\right)}, \end{array}$$
where, *α*_1_, *α*_2_, and *α*_3_ are the weight coefficients of intelligent health monitoring equipment, college students, and sports, respectively, and *ξ* is the adjustment error. The weight coefficient *ξ* is calculated from the data published by the National College Students' intelligent health monitoring organization [12].
(4) The health monitoring data of dynamic planning is mainly based on the statistical data of the National Center for Disease Control and Prevention. The intelligent health monitoring time is calculated as *T*, the evaluation results *θ*, and the simplification rate of health monitoring data = (monitoring data before processing − monitoring data after processing)/the total number of monitoring data obtained (100 m running, standing long jump, etc.) *∗* 100%. The specific formula is as follows:
  (3) $$\begin{array}{c} \iota =\left\|\frac{H\left(\cdot \right)-G_{i,j,k}}{G_{i}+G_{j}+G_{k}}\right\|•\left(\begin{array}{ccc} \alpha_{i} & 0 & 0\\ 0 & \alpha_{j} & 0\\ 0 & 0 & \alpha_{k} \end{array}\right)\cdot 100\text{\%,} \end{array}$$
where *G*_*i*,*j*,*k*_ is the intelligent monitoring data of *x*_*i*_, _,_*x*_*j*_, and *x*_*k*_, *G*_*i*_, *G*_*j*_, and *G*_*k*_ is the total amount of *x*_*i*_, *x*_*j*_, and *x*_*k*_, *H*(*·*) is the processed intelligent monitoring data, and $\left(\begin{array}{ccc} \alpha_{i} & 0 & 0\\ 0 & \alpha_{j} & 0\\ 0 & 0 & \alpha_{k} \end{array}\right)$ is the weight of the intelligent monitoring data in *x*_*i*_, *x*_*j*_, and *x*_*k*_.
(5) In order to improve the complex data (structured, semi-structured and unstructured) in college students' sports, realize the “intelligence” of the transformation between health monitoring data and reduce the error of initial monitoring data, subcontracting can be used for processing. Because the attribute of intelligent monitoring data is relatively simple, the Euclidean distance can be used for wavelet packet. First set the range of structured, unstructured, and semistructured monitoring data, and the formula is as follows:
  (4) $$\begin{array}{c} \left|S\right|=\frac{c_{l}}{\left(\sum_{l=0}^{n}c_{l}+\mu^{2}\right)}, \end{array}$$
where |*S*| is the Euclidean distance of each monitoring data; *c*_*l*_ is the intelligent; *c*_0_ is the initial cluster value; *μ* is the allowable error of clustering and is set by the power industry in the early stage of calculation, ∑_*l*=0_^*n*^*c*_*l*_ is the set of *c*_*l*_. According to formula (1) to formula (4) steps to calculate the conclusion, the dynamic programming algorithm uses the judgment matrix of wavelet function to subcontract the overall data. At the same time, sort the subcontracted data to form an orderly data flow. On this basis, the data processing capacity of dynamic programming method decreases exponentially. At the same time, the continuous tracking of dynamic programming algorithm increases the total amount of data, but the amount of data processing can be further improved by setting the subcontracting value. Therefore, the advantages of wavelet function and dynamic programming algorithm in data processing are very obvious.

RETRACTED

## 3. Build an Intelligent Health Monitoring Model Based on Dynamic Programming Algorithm

### 3.1. Construct the Relationship among College Students' Data Structure, Health Monitoring Impact, and Health Monitoring Dynamics

Intelligent health monitoring not only considers the monitoring accuracy of *x*_*i*_, *x*_*j*_, and *x*_*k*_ but also considers the synergy among them. Therefore, the relationship operator between *x*_*i*_, *x*_*j*_, and *x*_*k*_ should be constructed. It is assumed that the relationship between the three is divided into local fusion relationship (*x*_*i*_ and *x*_*j*_, *x*_*i*_ and *x*_*k*_, and *x*_*j*_ and *x*_*k*_) and overall fusion relationship (*x*_*i,*_*x*_*j,*_*x*_*k*_), which are expressed by *Pc* and *Pm*, respectively. Then, the calculation formula is as follows:

(5) $$\begin{array}{c} P_{\text{c}}\begin{array}{c} P_{\text{c}}=P_{m}\\ P_{c}\neq P_{m} \end{array}\overset{\text{location}}{\underset{\text{value}=1}{⇄}}P_{\text{m}}\left\{\begin{array}{c} P_{c_{0}}\\ \varphi \left(x\right)\frac{\left[\left(P_{c_{x_{i,j,k}}}-P_{\min}\right)\right.}{\bar{\sum \left.P_{c_{x_{i,j,k}}}-P_{\max}\right],}}\\ P_{m}\approx 0or1\\ P_{\max}\langle 1,P_{m}\rangle 1 \end{array}\right., \end{array}$$

where, *P*_*c*_0__ is local fusion, all fusion, *P*_min_ and *P*_max_ are the minimum *Pc* and *Pm* maximum values, which are set by local universities, and *φ*(*x*) is the fusion degree function of the above analysis, the value is between 0 and 1.

### 3.2. Construct the Accuracy Model of College Students' Intelligent Health Monitoring

Accuracy is the key index of intelligent health monitoring [13], and it is also the main purpose of dynamic programming algorithm optimization. Therefore, the accuracy operator should be constructed. The specific formula is as follows:

(6) $$\begin{array}{c} {\text{Inc}}_{l}{}^{o,p,q}=\left\{\begin{array}{c} 0<Inc_{l}{}^{o,p,q}<1\\ \begin{array}{c} \vec{\underset{\leftarrow }{{\text{Inc}}_{l}{}^{o,p,q}<\left\|\max\left[Inc_{l}{}^{n,n,n}\right]\right\|}}\\ \int_{I,j}^{n}\langle \left(\sum_{I=1}^{n}\max\left(Inc_{l}{}^{o,p,q}\right)\overset{\gg }{\underset{\ll }{⇄}}\min\left(Inc_{l}{}^{o,p,q}\right)\right)|||P_{c}\neq P_{m},P_{\max}\langle 1,\text{and}P_{m}\rangle 1\rangle \end{array} \end{array}\right.. \end{array}$$

Since the accuracy of *x*_*i,*_*x*_*j*_ and *x*_*k*_ is 0〈Inc_*l*_^*o*,*p*,*q*^〈1, 0〈Inc_*l*_^*o*,*p*,*q*^〈1 are required to shorten the range of max(Inc_*l*_^*o*,*p*,*q*^)⇄_≪_^≫^min(Inc_*l*_^*o*,*p*,*q*^) calculation accuracy. At the same time, the fusion error of the calculation results should be reduced, so $\prod \varphi \left(x\right)\lim_{l⟶\infty }\underset{0∼0.1}{\underset{⎵}{{∲}_{l}\sin\left(\alpha_{1,2,3}\right)}}$ should be between 0 and 0.1.

### 3.3. Calculation Steps of Operators in Intelligent Health Monitoring of College Students' Intelligent Equipment Devices

1. Build an intelligent health monitoring data set, *C*_*l*_ = {*c*_*1*_, *c*_*2*_,…, *c*_*i*_} and eliminate the intelligent monitoring data with digitization degree of <60%. Determine the weight coefficient and adjustment error according to the digital Economic Yearbook of power industry from 2015 to 2020;
2. The monitoring data *c*_*l*_ processed by wavelet function are processed structurally [14], semistructurally and unstructured to realize the “cleaning” of intelligent monitoring data.
3. Judge the fusion relationship of the monitoring data after “cleaning” and obtain the values of *Pc* and *Pm* of local and overall fusion relationships.
4. The iterative analysis of steps 1∼4 is carried out using MATLAB software, and the accuracy, calculation time, and effectiveness of the calculation results are output. The result are shown in Figure 3.

RETRACTED

## 4. The the Case Analysis of Intelligent Health Monitoring Based on Dynamic Programming Algorithm

### 4.1. The Actual Case Analysis

Taking college students in various regions as the research object, analyze the data structure *x*_*i*_ in intelligent equipment devices, the impact of intelligence on health monitoring *x*_*j*_, and the dynamics of health monitoring *x*_*k*_ as the input indicators. Local universities and national CDC provide *c*_0_  = 22.3, *μ*  = 0.02, *α*_0_  = 0.41, 100 iterations, and *P*_min_  = 0.23, *P*_max_  = 0.99. The specific monitoring data are shown in Table 1.

### 4.2. The Comparison of Data Processing Capacity of College Students' Intelligent Health Monitoring

The dynamic programming algorithm uses wavelet packet to preprocess the intelligent monitoring data [15], eliminate redundant monitoring data, and extract eigenvalues. The processing result is better than the static programming algorithm. The results are shown in Table 2.

It can be seen from Table 2 that the dynamic programming algorithm is consistent with the actual demand, while the monitoring data processing capacity of the static programming algorithm is quite different from the actual demand and does not change along the change of the actual demand curve. In the range of 0∼25 iterations, there is no significant difference in the processing capacity of monitoring data between the two algorithms, but there are significant differences in the range of 25∼50, 50∼75 and 75∼100 iterations, and the dynamic programming algorithm is better than the static programming algorithm, which is consistent with the results of relevant studies Wang [16]. With the increase of the number of iterations, the amount of monitoring data processing increases. The specific results are shown in Figure 4.

It can be seen from Figure 4 that in the monitoring stage of 0.6 years, the change range of dynamic programming algorithm is significantly less than that of static detection algorithm. Moreover, the processing capacity of dynamic programming algorithm is higher than the total data processing capacity. Therefore, the amount of data processing in dynamic programming algorithm is more reasonable. At same time, it can be seen from Figure 4 that the data processing capacity of dynamic programming is relatively stable without significant fluctuation, while the fluctuation of static programming algorithm is relatively large in the early stage and tends to be flat in the later stage, so the processing effect of dynamic programming is better, which is consistent with the results of relevant studies [17]. The comparison of the actual data processing capacity of the two methods is shown in Figure 5.

RETRACTED

As can be seen from Figure 5, the area of dynamic programming algorithm is significantly larger than that of static programming algorithm. Although the height of static programming algorithm is higher than that of dynamic algorithm, the overall area of dynamic programming algorithm is larger.

It can be seen from Figure 5 that the unit processing data of dynamic programming algorithm is significantly higher than that of static programming algorithm, which also fully explains the phenomenon that the processing process of dynamic programming algorithm is relatively stable. The main reason for the above problems is that the dynamic programming algorithm uses wavelet function for data subcontracting to reduce the complexity of data structure.

### 4.3. The Calculation Accuracy

The dynamic programming algorithm is used to analyze the data structure *x*_*i*_ in intelligent equipment devices, the impact of intelligence on health monitoring *x*_*j*_, and the results of the dynamic *x*_*k*_ of health monitoring. The results are shown in Table 3.

It can be seen from Table 3 that the data structure *x*_*i*_ in intelligent equipment devices of dynamic programming algorithm, the impact of intelligence on health monitoring *x*_*j*_, and the dynamic *x*_*k*_ accuracy and overall accuracy of health monitoring are better than those of static programming algorithm. It mainly understands that the planning algorithm integrates the weight coefficient and adjustment error, which is consistent with the results of relevant studies [18]. The above three indicators show small error changes in the dynamic planning algorithm, so as to avoid the interference of redundant monitoring data in the calculation and improve the accuracy of calculation. The results are shown in Figure 6.

As can be seen from Figure 6, the accuracy of dynamic programming algorithm is always higher than that of static algorithm, and the overall fluctuation range is small. The accuracy of dynamic programming algorithm is between 98% and 99%, whereas that of static programming algorithm is between 90% and 95%. Moreover, the stability of dynamic programming algorithm is better, which is significantly higher than that of static programming algorithm. The results are consistent with relevant domestic studies. The results are shown in Table 4.

RETRACTED

### 4.4. The Time of Intelligent Health Monitoring

It can be seen from Table 4 that the health monitoring processing time of dynamic planning algorithm is significantly less than that of static planning algorithm, and the whole health monitoring processing time is less than 25 s. According to the line segment slopes of the two algorithms, the health monitoring data of static planning show ups and downs, whereas the health monitoring data of dynamic planning change smoothly and the slope change range is small. This shows that the dynamic programming algorithm is better than the static programming algorithm, which can meet the requirements of intelligent health monitoring and also meet the standards of intelligent health monitoring by the ministry of health and local universities in 2021. The results are shown in Table 4.

As can be seen from Figure 7, the calculation time of dynamic programming method is always lower than that of static programming method, and the overall calculation time is almost the same. Therefore, the calculation time of dynamic programming is better. The variation range of calculation time of different algorithms is shown in Figures 8 and 9.

As can be seen from Figures 7 and 8, the variation range of calculation time of dynamic programming algorithm is significantly lower than that of static programming algorithm. This fully explains the problem of stable calculation time of dynamic programming algorithm and also shows that the data processing effect of dynamic programming algorithm is better. The variation range of dynamic programming algorithm is 0.9%, while that of static programming algorithm is 100%. Therefore, the result of dynamic programming algorithm is more stable and can be used in data processing of high-end intelligent devices.

## 5. Conclusion

By measuring the physical fitness of college students, evaluating the physical status and the effect of physical exercise, improving and urging the effective mechanism of college students to participate in physical exercise, scientifically guiding college students to carry out physical activities, so as to continuously enhance the physical fitness of college students, thus also providing effective national physical fitness monitoring data can be done. Intellectualization is the requirement of the ministry of health and local colleges and universities for college students in 2020, and it is also the direction of future development and reform of colleges and universities [19]. Since 2010, the intelligent development of College Students' monitoring has gradually increased. However, due to the large amount of monitoring data involved in equipment public, relevant specifications, and other links, the previous static planning Bayesian and genetic algorithms have achieved accurate evaluation, which affects the implementation of later improvement measures [20]. In this article, wavelet function and static programming method are combined to build a dynamic programming algorithm model to evaluate the intelligent health monitoring. The results show that the following: (1) intelligent wearable devices are popular among contemporary college students and play an important supporting role in college students' intelligent health monitoring. At the same time, due to the great pressure of study and work, college students are not only the main subhealth population in society but also the key health monitoring object. The dynamic programming algorithm constructed in this article can continuously monitor the health of college students and has the advantages of continuous and complete monitoring data. Dynamic programming monitoring can provide redundant data and solve the problem of data distortion in static programming. (2) The constructed model can effectively eliminate redundant monitoring data and accurately extract eigenvalues, which is consistent with the actual intelligent health monitoring requirements, and the calculation time is less than 25 s, and the evaluation process is stable. (3) Compared with static planning, the model is superior to static planning in terms of calculation accuracy. The accuracy of dynamic programming algorithm is between 98% and 99%, while that of static programming algorithm is between 90% and 95%. Moreover, the stability of dynamic programming algorithm is better, which is significantly higher than that of static programming algorithm. The results are consistent with relevant domestic studies. The monitoring data processing capacity and calculation time meets the standards of intelligent health monitoring by the ministry of health and local universities in 2021. The variation range of dynamic programming algorithm is 0.9%, while that of static programming algorithm is 100%. Therefore, the result of dynamic programming algorithm is more stable and can be used in data processing of high-end intelligent devices. Of course, this article has less research on the transmission technology and security technology of intelligent devices, and these contents are the guarantee of intelligence, so we will focus on the above two aspects in the future.

RETRACTED

## Figures and Tables

**Figure 1:** The monitoring proportion of intelligent equipment devices in different sports events from 2017 to 2021.

**Figure 2:** The intelligent equipment monitoring of intelligent equipment devices on College Students' sports events.

**Figure 3:** The Calculation flow of dynamic programming algorithm.

**Figure 4:** The processing capacity of intelligent health monitoring data at different times.

**Figure 5:** The data capacity of intelligent health monitoring at different times.

**Figure 6:** The calculation accuracy of different algorithms.

**Figure 7:** The calculation time of different algorithms.

**Figure 8:** The change range of dynamic programming algorithm calculates time.

**Figure 9:** The change range of static programming algorithm calculates time.

**Table 1:** The data sources of intelligent health monitoring of college students in actual cases.

Attribution area	Collection type	Collect content
Sports colleges and universities in Northeast China	ECG function monitoring, sleep quality, circulatory system	Big data, intelligent devices, cloud computing
Sports colleges and universities in North China	Subhealth, family history	Virtual simulation, smart client data collection
Physical education colleges and universities in Northwest China	Reproductive health, adolescent psychology, and blood health of female students	Intelligent device, mobile watch
Sports colleges and universities in Southeast China	Major genetic diseases and epidemic surveillance	Mobile hub, network platform
National Center for disease control and prevention	Prevention of sudden and serious diseases	Mobile phone, Big data
Private health monitoring organization	Sub ealth, blood pressure, blood lipid	University network platform
World health organization	Epidemic diseases, major diseases, and sudden diseases	QQ chatting software, VR game, Bluetooth headset big data,

Note: the monitoring data comes from the data of the National Center for Disease Control and prevention from 2015 to 2020. The choice of collection type and attribution area is based on the relevant literature at home and abroad and the actual survey results.

**Table 2:** The average processing capacity of monitoring data of different algorithms.

Different methods	Iteration number range (times)	Average monitoring data processing capacity (km)
Dynamic programming algorithm	0∼25	32.32 ± 2.32^*∗∗*^

Standing long jump, 50-m sprint, 1000-vm long run, basketball	25∼50	48.62 ± 3.28^*∗*^
	50∼75	65.28 ± 4.02^*∗*^
	75∼100	82.23 ± 1.23^*∗*^

Total processing capacity		228.45 ± 3.22^*∗*^

Static programming algorithm	0∼25	22.37 ± 1.32

Standing long jump, 50-m sprint, 1000-m long run, basketball	25∼50	40.31 ± 4.16
	50∼75	55.08 ± 4.32
	75∼100	72.13 ± 1.82

Total processing capacity		189.89 ± 4.12

Compared with static programming algorithm, ^*∗*^*P* < 0.05, ^*∗∗*^*P* > 0.05.

RETRACTED

**Table 3:** The accuracy of different algorithms.

The different methods	The evaluating indicator	The accuracy rate (%)
The dynamic programming algorithm	*x*_*i*_	98.23^*∗*^
	*x*_*j*_	99.23^*∗*^
	*x*_*k*_	97.62^*∗*^

The total accuracy		98.32

The static programming algorithm	*x*_*i*_	92.32
	*x*_*j*_	96.23
	*x*_*k*_	95.72

The total accuracy		95.98

Compared with static programming algorithm, ^*∗*^*P* < 0.05; The value range is 0∼100.

**Table 4:** The calculation time of different algorithms.

The different methods	The calculation time (seconds)
The dynamic programming algorithm	82.32
The static programming algorithm	81.22

Note: the value range is 0∼100.

## Data Availability

The data used to support the ﬁndings of this study are available from the corresponding author upon request.
